The article "Prediction of Severe Injury in Bicycle Rider Accidents: A Multicenter Observational Study" was published in 2022. Journal: Emerg Med Int.

# Prediction of Severe Injury in Bicycle Rider Accidents: A Multicenter Observational Study

**DOI:** 10.1155/2022/7994866

**Published:** 2022-05-27

**Authors:** Il-Jae Wang, Young Mo Cho, Suck Ju Cho, Seok-Ran Yeom, Sung Wook Park, So Eun Kim, Jae Chol Yoon, Yeaeun Kim, Jongho Park

**Affiliations:** ^1^Department of Emergency Medicine, Pusan National University School of Medicine and Biomedical Research Institute, Pusan National University Hospital, Busan, Republic of Korea; ^2^Department of Emergency Medicine, Jeonbuk National University Hospital, Jeonju, Republic of Korea; ^3^Department of Health Care Management, Catholic University of Pusan, Busan, Republic of Korea; ^4^Division of Health Administration, Gwangju University, Gwangju, Republic of Korea

## Abstract

**Introduction:**

This study aimed to establish a predictive model that includes physiological parameters and identify independent risk factors for severe injuries in bicycle rider accidents.

**Methods:**

This was a multicenter observational study. For four years, we included patients with bicycle rider injuries in the Emergency Department-Based Injury In-depth Surveillance database. In this study, we regarded ICD admission or in-hospital mortality as parameters of severe trauma. Univariate and multivariate logistic regression analyses were performed to assess risk factors for severe trauma. A receiver operating characteristic (ROC) curve was generated to evaluate the performance of the regression model.

**Results:**

This study included 19,842 patients, of whom 1,202 (6.05%) had severe trauma. In multivariate regression analysis, male sex, older age, alcohol use, motor vehicle opponent, load state (general and crosswalk), blood pressure, heart rate, respiratory rate, and Glasgow Coma Scale were the independent factors for predicting severe trauma. In the ROC analysis, the area under the ROC curve for predicting severe trauma was 0.848 (95% confidence interval: 0.830–0.867).

**Conclusion:**

We identified independent risk factors for severe trauma in bicycle rider accidents and believe that physiologic parameters contribute to enhancing prediction ability.

## 1. Introduction

Bicycles are gaining popularity because of their accessibility for people of all ages and their versatility in use for exercise and transportation [1]. According to data reported in 2004, the number of cyclists worldwide is estimated to be approximately 800 million [2]. Recently, as individual sports have received increasing attention due to the prolonged coronavirus-19 pandemic, the number of bicycle users is rapidly increasing [3, 4]. As bicycles reduce traffic congestion and environmental pollution and benefit public health, many countries recommend using bicycles as a national strategy [4–6]. In Korea, national efforts, such as revising traffic laws, expanding bicycle-only roads, and public relations activities, have been implemented. In 2016, the number of bicycle users was estimated to be approximately 13 million [7, 8].

However, the number of patients with bicycle-related injuries has also increased in concordance with the increase in the number of cyclists. Previous research has shown that riding a bicycle presents a risk of death 12 times higher than that of driving a car [9, 10]. In Korea, bicycle accidents are increasing yearly, and the proportion of bicycle accident fatalities among all traffic fatalities is also increasing [7, 11]. Predicting patients severely injured while using bicycles is crucial for improving management and establishing preventive policies. Several previous studies have evaluated the risk factors for cyclist injuries, including demographic characteristics (age and sex), behavioral factors (alcohol use and helmet use), and environmental factors (road type, time and season of injury, and injury opponent) [12–16]. However, few studies have assessed risk factors, including physiological parameters (blood pressure, mentality, and respiratory rate).

The purpose of our study was to establish a predictive model that includes physiological parameters and identify independent risk factors for severe injuries in bicycle rider accidents.

## 2. Materials and Methods

### 2.1. Study Design and Setting

This was a retrospective multicenter observational study performed using the Emergency Department-Based Injury In-depth Surveillance (EDIIS) database of Korea. The EDIIS is a nationwide database that includes all injured patients who presented to the emergency department throughout Korea. The Korea Centers for Disease Control and Prevention (KCDC) established the EDIIS in 2006, with data collected from five hospitals. The number of participating hospitals has steadily increased, with 23 hospitals currently participating in the EDIIS. The EDIIS aims to produce statistics on risk factors and consequences related to injury occurrence as well as provide helpful information for developing injury prevention and management policies.

The study complied with the principles of the Declaration of Helsinki. The institutional review board of our institution approved the study protocol. Patient information was anonymously analyzed; as such, the requirement for informed consent was waived.

We included patients with bicycle rider injuries in the EDIIS database for four years (between 2016 and 2019). The exclusion criteria were as follows: age <15 years, cardiac arrest when presented to the ED, and transferred to other hospitals. The following data were extracted from the database: sex, age, alcohol use, season of injury, time of injury, use of helmet, injury opponent, injury location, systolic blood pressure (SBP), diastolic blood pressure (DBP), pulse rate (PR), respiratory rate (RR), Glasgow Coma Scale (GCS), intensive care unit (ICU) admission, and in-hospital mortality. The time of injury was classified into three groups: day (08 : 00–15 : 59), evening (16 : 00–23 : 59), and night (00 : 00–7 : 59). Injury opponents were classified into four groups: pedestrians, bicycles, motor vehicles, and others. Injury locations were classified into four groups: general roads, bicycle lanes, crosswalks, and others. In this study, we regarded ICU admission or in-hospital mortality as parameters of severe trauma.

### 2.2. Statistical Analysis

Data analysis was performed using IBM SPSS version 26 (IBM Corp., Armonk, New York, USA). We completed the Shapiro–Wilk test for continuous variables, and none of the continuous variables showed a Gaussian distribution. Continuous variables are presented as medians and interquartile ranges. Categorical variables are presented as frequencies (percentages). Continuous variables were compared using the Wilcoxon rank-sum test, and categorical variables were compared using Fisher's exact test. Continuous variables were compared using the Mann–Whitney *U* test, and categorical variables were compared using Fisher's exact test. Statistical significance was set at *P* < 0.05.

Univariate and multivariate logistic regression analyses were performed to assess risk factors for severe trauma. All significant variables in the univariate analysis were subjected to multivariate logistic regression analysis. All variables with a *P* value of less than 0.05 were included in a logistic regression analysis. To evaluate the performance of the multivariate logistic regression model, a receiver operating characteristic (ROC) curve was generated, and the area under the receiver operating characteristics curve (AUROC) was calculated. SPSS version 26.0 (SPSS Inc., Chicago, IL, USA) was used for the statistical analysis.

## 3. Results

### 3.1. Patient Characteristics

During the study period, 28,812 patients injured due to bicycle riding were registered in the EDIIS registry. The exclusion criteria were as follows: age <15 years (*n* = 8155), cardiac arrest when presented to the ED (*n* = 3), and transfer to other hospitals (*n* = 812). A total of 8,970 patients were excluded. The final study population included 19,842 patients.

Among all patients, 15,242 (76.8%) were male and 4,600 (23.2%) were female, with a median age of 47 (27–60) years. A total of 1,202 (6.05%) patients had severe trauma. We compared the characteristics of patients in the severe and nonsevere trauma groups. Patients in the severe trauma group were significantly older (*P* < 0.001), were predominantly male (*P* < 0.001), drank significantly more alcohol, and displayed lower helmet use rates, lower GCS scores, and lower SBP. Furthermore, the time of injury, season of injury, injury location, and injury opponent showed significant differences between the two groups.  Table 1 provides the characteristics of the study population.

### 3.2. Univariate and Multivariate Logistic Regression and ROC Analysis

Univariate analysis revealed significant differences in male sex, age, alcohol use, season (fall and winter), time of day (evening and nonevening), motor vehicle opponent, load state (general, crosswalk, and bicycle road), nonhelmet use, SBP, HR, RR, and GCS (Table 2). In the multivariate analysis, differences in male sex, older age, alcohol use, motor vehicle opponent, load state (general and crosswalk), SBP, HR, RR, and GCS were independent predictors of severe trauma (Table 3). ROC analysis was performed, and AUROCs were calculated to assess the predictive value of the multivariate logistic regression model for severe trauma. The AUROC for predicting severe trauma was 0.848 (95% confidence interval, 0.830–0.867) (Figure 1).

## 4. Discussion

This study was designed to identify the risk factors for severe trauma in patients presenting with bicycle riding injuries. We found that male sex, older age, alcohol use, motor vehicle opponent, load state (general and crosswalk), SBP, HR, RR, and GCS score were independent risk factors. The bicycle road, nonhelmet use, season (fall and winter), and evening time of day were statistically significant in the univariate regression analysis but not in the multivariate analysis. The AUROC value of the multivariate regression model was 0.848, indicating excellent predictive power [17].

Among the independent risk factors identified in our study, older age, male sex, and alcohol use were consistent with previous studies [11, 15, 16, 18]. The male sex is known to be at risk of severe trauma and has more frequent accidents than women; in our study, the frequency of accidents was approximately three times higher in men. It can be assumed that men drive less safely than women, and, on average, men are heavier and therefore have greater kinetic energy [16]. As age increased, the likelihood of severe trauma increased. A previous study reported that drivers aged ≥50 years were more than twice as likely to have severe injuries as the youngest group. Shin et al. reported that the hospitalization rate increased with increasing age [15, 19]. In this study, excluding children, when age was considered as a continuous variable, the adjusted OR was 1.038 (95% confidence interval, 1.032–1.044, *P* < 0.001). This may be due to a decrease in exercise capacity, bone density, and muscle mass, caused by aging and various underlying diseases [19].

Recently, two studies related to drinking in bicycle accidents have been conducted in Korea. Seo et al. revealed that the rate of severe injury in the alcohol intake group was more than double among cyclists, and Jeong et al. showed that the alcohol intake group was less likely to wear protective gear, leading to a higher risk of traumatic brain injuries [11, 20].

Similarly, drinking was significantly higher in patients with severe injury outcomes in this study. Multivariate logistic regression was used to identify independent risk factors for severe injury. Although the drinking rate reported in this study was relatively lower than that in Germany and the United States, institutional and educational initiatives are needed to reduce the drinking rate among cyclists [21, 22].

Significantly, our findings showed that accidents at crosswalks are more likely to lead to severe clinical outcomes. This finding is surprising, given that crosswalks are generally considered safe. It has been demonstrated that accidents at crosswalks are prevalent, and the injury severity of patients varies depending on the type of crosswalk [23, 24]. However, because these studies were conducted on pedestrians while crossing the road and highlighted their safety, further research that focuses specifically on cyclists is needed to understand the injury severity in this population.

The analysis for predicting the injury severity of bicycle accidents has been conducted using different risk factors and analytical techniques [13, 15]. To the best of our knowledge, this is the first study to include physiological parameters, such as BP, HR, RR, and GCS, as predictors of bicycle injury. Since the AUROC value from the multivariate regression was relatively high (0.84), it seems reasonable to conclude that these physiological parameters contribute to the prediction of injury severity.

Our study has some limitations. First, it was a retrospective study. Therefore, potential bias could not be completely excluded. Second, although EDIIS is a multicenter, nationwide system, EDs that joined EDIIS were relatively high-level EDs. Therefore, the patients included in this study may not represent all cases of bicycle rider crashes. Third, because EDIIS contains only predefined variables, potentially useful variables, such as prehospital vital signs, helmet types, or whether to use goggles, cannot be used. It might imply the need for extended and in-depth variables about injured patients.

## 5. Conclusions

This study identified that male sex, older age, alcohol use, motor vehicle opponent, load state (general and crosswalk), SBP, HR, RR, and GCS were the independent factors for the prediction of severe trauma in bicycle riders injured due to accidents. The AUROC of our multivariate regression model showed excellent predictive power. We believe that our findings will contribute to better triage and improved policies for patients with bicycle rider crashes.

## Figures and Tables

**Figure 1:** Multivariate logistic regression ROC curve.

**Table 1:** General characteristics according to the clinical outcome at discharge.

Variables	Total (*n* = 19,842)	Nonsevere outcome(*n* = 18,640; 93.9%)	Severe outcome (including death)(*n* = 1,202; 6.1%)	*P* value
Sex, *n* (%)				0.000
Male	15,242 (76.8)	14,228 (76.3)	1,014 (84.4)	
Female	4,600 (23.2)	4,412 (23.7)	188 (15.6)	
Age (y), median (IQR)	47 (27–60)	45 (26–59)	63 (50–74)	0.000
Drinking, *n* (%)				0.000
No	18,567 (93.6)	17,478 (93.8)	1,089 (90.6)	
Yes	1,275 (6.4)	1,162 (6.2)	113 (9.4)	
Season, *n* (%)				0.000
Spring	5,305 (26.7)	5,027 (27.0)	278 (23.1)	
Summer	6,636 (33.5)	6,283 (33.7)	353 (29.4)	
Fall	5,812 (29.3)	5,419 (29.0)	393 (32.7)	
Winter	2,089 (10.5)	1,911 (10.3)	178 (14.8)	
Time, *n* (%)				0.000
Day	7,800 (39.3)	7,269 (39.0)	531 (44.2)	
Evening	8,867 (44.7)	8,406 (45.1)	461 (38.4)	
Night	3,175 (16.0)	2,965 (15.9)	210 (17.5)	
Opponent party, *n* (%)				0.000
Pedestrian	166 (1.0)	159 (1.0)	7 (0.7)	
Bicycle	738 (4.6)	723 (4.8)	15 (1.5)	
Vehicle	4,743 (29.4)	4,150 (27.4)	593 (61.5)	
Others	10,492 (65.0)	10,142 (66.8)	350 (36.3)	
Place, *n* (%)				0.000
General road	8,152 (57.9)	7,528 (56.8)	624 (75.3)	
Cross walk	315 (2.2)	280 (2.2)	35 (4.2)	
Bicycle lane	1,676 (12.0)	1,646 (12.4)	30 (3.6)	
Others	3,931 (27.9)	3,791 (28.6)	140 (16.9)	
Protection equipment, *n* (%)				0.000
No	14,378 (78.4)	13,493 (78.0)	885 (84.4)	
Yes	3,968 (21.6)	3,805 (22.0)	163 (15.6)	
SBP, median (IQR)	137 (121–151)	137 (122–151)	134 (115–155)	0.000
DBP, median (IQR)	80 (71–90)	80 (71–90)	80 (70–91)	0.046
HR, median (IQR)	81 (73–91)	81 (73–90)	83 (72–96)	0.001
RR, median (IQR)	20 (18–20)	20 (18–20)	20 (18–20)	0.000
GCS, median (IQR)	15 (15–15)	15 (15–15)	15 (7–15)	0.000

IQR, interquartile range; SBP, systolic blood pressure; DBP, diastolic blood pressure; HR, heart rate; RR, respiratory rate; GCS, Glasgow Coma Scale.

**Table 2:** Association between severe outcome and other variables using univariate logistic regression.

Variables	Severe outcome (including death)			
	OR	95% CI		*P* value
Sex				
Female	1			
Male	1.673	1.426	1.961	0.000
Age (y)	1.043	1.039	1.046	0.000
Drinking				
No	1			
Yes	1.561	1.275	1.911	0.000
Season				
Spring	1			
Summer	1.016	0.864	1.194	0.848
Fall	1.311	1.119	1.536	0.001
Winter	1.684	1.385	2.048	0.000
Time				
Night	1			
Day	1.031	0.874	1.217	0.714
Evening	0.774	0.654	0.916	0.003
Opponent party				
Others	1			
Pedestrian	1.276	0.594	2.740	0.532
Bicycle	0.601	0.357	1.014	0.056
Vehicle	4.141	3.611	4.748	0.000
Place				
Others	1			
General road	2.245	1.861	2.707	0.000
Crosswalk	3.385	2.292	4.998	0.000
Bicycle lane	0.494	0.331	0.375	0.001
Protection equipment				
Yes	1			
No	1.531	1.291	1.816	0.000
SBP	0.993	0.990	0.996	0.000
DBP	0.995	0.991	0.999	0.018
HR	1.013	1.009	1.017	0.000
RR	1.062	1.131	1.195	0.000
GCS	0.449	0.416	0.485	0.000

SBP, systolic blood pressure; DBP, diastolic blood pressure; HR, heart rate; RR, respiratory rate; GCS, Glasgow Coma Scale; OR, odds ratio; CI, confidence interval.

**Table 3:** Association between severe outcome and other variables using multivariate logistic regression.

Variables	Severe outcome (including death)			
	OR	95% CI		*P* value
Sex				
Female	1			
Male	1.431	1.099	1.863	0.008
Age (y)	1.038	1.032	1.044	0.000
Drinking				
No	1			
Yes	1.521	1.091	2.120	0.013
Season				
Spring	1			
Summer	0.953	0.729	1.246	0.726
Fall	1.239	0.954	1.609	0.108
Winter	1.139	0.813	1.595	0.450
Time				
Night	1			
Day	1.319	0.977	1.780	0.071
Evening	1.300	0.966	1.750	0.084
Opponent party				
Others	1			
Pedestrian	1.616	0.567	4.607	0.370
Bicycle	0.568	0.277	1.163	0.122
Vehicle	2.412	1.951	2.982	0.000
Place				
Others	1			
General road	1.316	1.026	1.688	0.030
Cross walk	1.848	1.091	3.129	0.022
Bicycle lane	0.657	0.393	1.098	0.109
Protection equipment				
Yes	1			
No	1.162	0.893	1.510	0.263
SBP	0.982	0.976	0.987	0.000
DBP	0.998	0.989	1.007	0.624
HR	1.010	1.004	1.017	0.002
RR	1.061	1.031	1.091	0.000
GCS	0.507	0.469	0.548	0.000

SBP, systolic blood pressure; DBP, diastolic blood pressure; HR, heart rate; RR, respiratory rate; GCS, Glasgow Coma Scale; OR, odds ratio; CI, confidence interval.

## Data Availability

Data cannot be shared publicly because the data are owned by the Korea Centers for Disease Control and Prevention (CDC). Data are available after the review of the letter of data request for researchers who meet the criteria for access to confidential data.
